# The Correlation between ^18^F-FDG PET/CT Imaging SUVmax of Preoperative Colon Cancer Primary Lesions and Clinicopathological Factors

**DOI:** 10.1155/2021/4312296

**Published:** 2021-09-17

**Authors:** Dacheng Li, Ying Wang, Weili Liu, Qiusong Chen, Li Cai, Xiling Xing, Shuo Gao

**Affiliations:** ^1^Department of PET-CT Diagnostic, Tianjin Medical University General Hospital, Tianjin 300052, China; ^2^Department of Nuclear Medicine, The Affiliated Hospital of Qingdao University, Qingdao 266000, Shandong Province, China; ^3^Interventional Operation Room, The Affiliated Hospital of Qingdao University, Qingdao 266000, Shandong Province, China

## Abstract

**Background:**

The purpose of this study is to explore the correlation between the ^18^F-FDG PET/CT imaging maximum standardized uptake value (SUVmax) of preoperative colon cancer primary lesions and clinicopathological factors.

**Methods:**

88 colon cancer patients diagnosed by histopathology were collected from January 2014 to December 2015. ^18^F-FDG PET/CT imaging was performed before surgery. Kaplan–Meier survival analysis was used to assess the prognosis of colon cancer patients.

**Results:**

The ^18^F-FDG PET/CT imaging SUVmax value of preoperative colon cancer primary lesion was significantly correlated with the length of the lesion, clinical stage, histopathological type, and the degree of tumor differentiation. The SUVmax value of tumors with long-diameter, ≥ 3 cm, clinically high-stage, adenocarcinoma, and poorly differentiated lesions was significantly high. In addition, the consistency between PET/CT and surgical pathological results at stage I and IV was higher. Stage II and III PET/CT are basically consistent with the pathological results of surgery. Kaplan–Meier survival analysis showed that the 5-year event-free survival rate of the SUVmax > 18.26 group was significantly lower than that of the SUVmax ≤ 18.26 group.

**Conclusion:**

^18^F-FDG PET/CT imaging SUVmax of preoperative colon cancer primary lesions can not only reflect the proliferation and invasion ability but also monitor the recurrence and metastasis of colon cancer.

## 1. Introduction

The incidence of colon cancer ranks third among malignant tumors, and its mortality rate is second only to lung cancer, liver cancer, and gastric cancer. Colon cancer is a serious threat to human life and health [1]. With the changes in people's dietary habits and the intensification of population aging, the incidence and mortality of colon cancer in China have shown a continuous upward trend in recent years. In addition, the incidence of colon cancer has risen to the second place among gastrointestinal malignancies [2]. The main method of treating early colon cancer is surgical resection. Postoperative patients with advanced colon cancer have a certain rate of recurrence and metastasis. Therefore, early diagnosis and accurate preoperative evaluation of clinicopathological factors are key factors that guide the treatment and prognosis of colon cancer patients.

Currently, traditional imaging examination methods include CT and MRI. They judge the lesion based on the anatomical shape of the lesion. Sometimes, it is difficult to distinguish between benign and malignant lesions. There are limitations in judging lymph node or distant metastasis [3]. PET/CT combines the advantages of PET and CT. PET can display the pathophysiological function of malignant tumor lesions. CT can accurately display the anatomical structure. PET/CT can realize the same machine fusion of morphological and functional imaging. In addition, PET/CT not only makes up for the deficiencies of CT qualitative difficulties and inaccurate PET positioning but also greatly improves the diagnostic efficiency of malignant tumors [4]. PET/CT has unique advantages over traditional imaging in monitoring the recurrence, metastasis, and prognosis of colon cancer [5]. The maximum standardized uptake value (SUVmax) is a semiquantitative index of PET/CT. Understanding the correlation between SUVmax and clinicopathological factors can further guide clinical treatment and evaluate prognosis.

In this study, preoperative ^18^F-FDG PET/CT imaging data of 88 colon cancer patients were retrospectively analyzed to evaluate the correlation between SUVmax and clinicopathological factors. This study can provide the basis for guiding the treatment and prognostic follow-up of colon cancer.

## 2. Materials and Methods

### 2.1. Patients

88 patients with colon cancer diagnosed by histopathology participated in our research. ^18^F-FDG PET/CT imaging was performed before surgery. Surgery or colonoscopy histopathological examination was performed within 2 weeks after PET/CT examination. Clinical stage refers to the TNM staging standard for colon cancer proposed by the American Joint Committee on Cancer (AJCC) and the Union for International Cancer Control (UICC) [6]. The clinicopathological factors of 88 patients with colon cancer are shown in Table 1.

### 2.2. Inclusion and Exclusion Criteria

Inclusion criteria: ① All patients were diagnosed for the first time and were cancers of the colon primary site. ② All patients had not received antitumor treatment within half a year before the examination. ③ All patients underwent ^18^F-FDG PET/CT examination before operation. ④ All patients and their families in this study signed informed consent.

Exclusion criteria: ① patients with other malignant tumors; ② pregnant, breastfeeding, or diabetic patients; and ③ patients with incomplete data.

### 2.3. PET/CT Examination

Before the examination, the patient fasted for 4–6 hours. Fasting blood glucose should be maintained below 7.1 mmol/L. After injecting 18 F-FDG into the elbow vein at a dose of 4.0 MBq/kg, the patient rested quietly for 50–60 minutes. After the patient has passed the urine, a regular PET/CT scan (from the top of the skull to the middle of the femur) was performed. If necessary, the lower limbs or soles of the feet were also scanned. Then, 6∼8 beds were collected (3 min/bed). The tube voltage and tube current are 120 kV and 150 mA, respectively. The layer thickness is 3.75 mm. Three-dimensional acquisition is performed during the PET scan, and the layer thickness is 3.25 mm. The CT data are used for attenuation correction, and the maximum expected value iteration method of ordered subsets is used for image reconstruction. The reconstruction data are uploaded to the AW4.5 workstation for image display and data processing.

### 2.4. Image Analysis

Two experienced nuclear medicine physicians observe and analyze each PET/CT image. When the diagnosis is inconsistent, the result after discussion by 2 or more nuclear medicine doctors shall prevail. Semiquantitative analysis is used to select the layer with the highest radioactive concentration of the lesion to delineate the region of interest (ROI). Also, the system automatically measures the SUVmax of the lesion.

### 2.5. PET/CT Preoperative Stage Standard

PET/CT preoperative staging is based on the TNM staging system for colon cancer proposed by the American Joint Committee on Cancer (AJCC), the Union for International Cancer Control (UICC) [6], and other PET studies [7].

T0: no primary tumor was found.

T1∼T2: the lumen is locally thickened, but the outer wall is still smooth. The fat spaces around is still clear. Also, the radioactivity of the lesion was concentrated on the PET image (SUVmax ≥ 2.5).

T3: the tube wall is locally thickened, and the lumen is obviously narrowed. The shape of the tube wall is irregular and uneven. The fat gap is not clear and fuzzy. The primary focus and the main lesions and affected organs or tissues show radioactivity concentration on the PET image.

T4: the tumor breaks through the serosal layer, and the tube wall thickens more obviously. Also, the lumen becomes narrower. The density of peripheral fat interstices is increased, which invades the structure of adjacent organs. The mass and the invaded organs showed radioactivity concentration on the PET image.

N0: no regional lymph node metastasis was found.

N1: there are 1 to 3 regional lymph node metastases. CT shows that the long diameter of the lymph node is >1.0 cm. The long diameter is less than 1.0 cm, but SUVmax ≥ 2.0.

N2: there are more than 4 regional lymph node metastases.

M0: no distant metastasis was found.

M1: distant metastasis was exhibited. The PET image of the metastasis shows the radioactivity concentration. Also, the shadow of the lesion can be seen on CT.

### 2.6. Follow-Up and Prognostic Evaluation

After initial treatment (surgery, radiotherapy, and chemotherapy), 88 patients with colon cancer were followed up by a combination of outpatient review, telephone, and electronic medical record system. The follow-up end point was December 2020. The follow-up time was 3–60 months (1 time/3–6 months).

The patients received CT, ^18^F-FDG PET/CT and colonoscopy regularly. The occurrence of recurrence, new metastasis, or death is defined as an “event.” Event-free survival refers to the absence of recurrence, new metastasis, or death from the end of initial treatment to the end of follow-up.

### 2.7. Statistical Analysis

The data were analyzed using SPSS 22.0. Data are expressed as mean ± SD. The independent sample *t*-test was used to compare the average SUVmax between the two groups. PET/CT was calculated to determine the sensitivity, specificity, accuracy, positive predictive value (PPV), and negative predictive value (NPV) of colon cancer clinical stage. The kappa test was used to evaluate the consistency of PET/CT in the preoperative clinical stage and pathological diagnosis. Kappa value < 0.4 indicates that the consistency of the test results is poor. The kappa value is generally consistent between 0.4 and 0.75. Kappa value > 0.75 means higher consistency. The Kaplan–Meier method and log-rank test were used for survival analysis. *P* < 0.05 indicates that the difference is statistically significant.

## 3. Results

### 3.1. Uptake of 18 F-FDG in Primary Lesions and Metastases

Eighty-eight colon cancer lesions uptake 18 F-FDG significantly. As shown in Figure 1, the sigmoid colon cancer lesions significantly uptake FDG, and the SUVmax was about 37.6. The SUVmax of peri-intestinal metastases was about approximately 8.4.  Figure 2 shows that the SUVmax of colon cancer was about 17.0. The size of the enlarged lymph node next to the right colon was about 10*∗*11 mm, and the SUVmax was about 4.6.  Figure 3 showed sigmoid colon cancer (SUVmax, 20.5) with multiple lung metastases (SUVmax, 15.3).

### 3.2. The Correlation between ^18^F-FDG PET/CT Imaging SUVmax Value before Colon Cancer Surgery and Clinicopathological Factors

The ^18^F-FDG PET/CT imaging lesion SUVmax of colon cancer before surgery was not significantly correlated with the patient's gender, age, and tumor location (*P* > 0.05, Table 2). But, it was closely related to the length of the lesion, clinical stage, histopathological type, and the degree of tumor differentiation (*P* < 0.01, Table 2). The SUVmax value of tumor with long-diameter, ≥ 3 cm, clinically high-stage, adenocarcinoma, and poorly differentiated lesions was significantly higher than that of short-diameter, <3 cm, clinically low-stage, mucinous adenocarcinoma, and well-differentiated tumor lesions (*P* < 0.01, Table 2).

### 3.3. Comparison of Clinical Stage Judged by ^18^F-FDG PET/CT Imaging and the Pathological Stage

Taking pathological diagnosis as the gold standard, the pathological stage results of 88 colon cancer patients and the sensitivity, specificity, accuracy, PPV, NPV, and kappa value of PET/CT stage are shown in Table 3. The consistency between PET/CT and surgical pathological results at stage I and IV was high (kappa = 0.789, 1.000; *P* < 0.05). The consistency between PET/CT and surgical pathological results at stage II and III was moderate (kappa = 0.553, 0.722; *P* < 0.05).

### 3.4. The Effect of the ^18^F-FDG PET/CT Imaging SUVmax Value of Primary Colon Cancer before Surgery on the Prognosis of Patients

Kaplan–Meier survival analysis showed that the 5-year event-free survival rate of the ^18^F-FDG PET/CT imaging SUVmax > 18.26 group (preoperative primary colon cancer) was significantly lower than that of the SUVmax ≤ 18.26 group (*x*^2^ = 14.363, *P* < 0.01, Figure 4).

## 4. Discussion

Colon cancer is one of the common malignant tumors of the digestive system, which can easily cause metastasis. When colon cancer has lymph node metastasis, the 5-year survival rate of the patients drops from 75% to about 30% [8]. Therefore, it is very important to conduct accurate clinicopathological factors analysis before colon cancer surgery. In addition to clarifying the location, size, and nature of the tumor lesions before surgery, it is also necessary to clarify the biological behaviors such as the extent of local infiltration, clinical stage, and the degree of lesion differentiation. Accurate analysis of clinicopathological factors can guide individualized treatment and optimize the treatment plan for colon cancer patients. It also reduces the risk and complications of blind surgery and improves the prognosis of patients [9].

At present, imaging examination has become one of the main methods for preoperative diagnosis of cancer lymph node metastasis. Compared with other imaging methods, CT has the characteristics of high sensitivity and specificity in judging lymph node metastasis, low false positive rate, less trauma to patients, and economical benefits [10]. Malignant tumor cells have active metabolism and high level of glycolysis. 18 F-FDG uptake increases and accumulates in cells. For small lesions, PET/CT may detect slight metabolic changes at an early stage [11]. PET/CT imaging can detect lesions early and immediately observe tumor cell proliferation and metabolic changes [9]. ^18^F-FDG PET/CT uses a semiquantitative index SUV to reflect the metabolism of the lesion. Also, the morphological changes of the lesions are observed by CT. ^18^F-FDG PET/CT can distinguish the nature of lesions together [12]. ^18^F-FDG PET/CT is suitable for patients of all ages, especially those who cannot undergo colonoscopy. In addition, ^18^F-FDG PET/CT plays an important role in tumor localization, staging, efficacy monitoring, and detection of distant metastases. In recent years, ^18^F-FDG PET/CT has gradually been used to assess the preoperative clinicopathological factors of colon cancer [13]. ^18^F-FDG PET/CT realizes the simultaneous fusion of functional metabolic imaging and anatomical morphology imaging. One imaging can simultaneously display the distribution, morphology, and metabolic status of multiple organs throughout the body. Its advantages in tumor diagnosis, stage, efficacy evaluation, and prognosis prediction are also increasingly prominent.

PET/CT uses SUV to measure the uptake of 18 F-FDG by colon cancer lesions, and SUVmax is usually used as an evaluation index. Analyzing the correlation between SUVmax and patients' clinicopathological factors is crucial to formulating preoperative treatment plans. This study showed that SUVmax was significantly related to lesion length, clinical stage, pathological type, and histological differentiation. Mucinous adenocarcinoma lesions require less ^18^F-FDG due to more mucus. Adenocarcinoma, especially poorly differentiated adenocarcinoma, has many malignant cells and high levels of metabolism. Therefore, adenocarcinoma requires more 18 F-FDG [14], which has a higher SUVmax value. In this study, the SUVmax of poorly differentiated and adenocarcinoma lesions was significantly higher than that of well-differentiated and mucinous adenocarcinoma. Accurately judging the clinical stage before surgery is particularly critical for guiding the choice of surgical plan. The National Comprehensive Cancer Network (NCCN) diagnosis and treatment guidelines proposed that neoadjuvant radiotherapy and chemotherapy should be performed for patients at stage III and IV to reduce the recurrence rate after surgery. Patients at stage I and II can be directly operated on [15]. The size of the lesion reflects the proliferation ability of the tumor. The invasion of surrounding tissues, lymph nodes, or distant metastasis reflects the tumor's invasion ability. In this study, the SUVmax value of tumor lesions with a long diameter, ≥ 3 cm, was significantly higher than that of tumor lesions with a short diameter, less than 3 cm. Lymph node metastasis is the most common way of colon cancer metastasis [16]. Approximately 20% of newly diagnosed colon cancer patients have distant metastases [17]. The most common site of metastasis is the liver. The number and location of liver metastases will affect the choice of surgical methods [18]. Previous studies have shown that the distant metastases accuracy of CT detection varies greatly, ranging from 55% [19] to 100% [15]. The sensitivity of PET/CT to distant metastases is higher than that of CT and MRI [20]. In this study, the consistency of between PET/CT and surgical pathological results at stage I and IV was high, and the consistency of between PET/CT and surgical pathological results at stage II and III was moderate. Therefore, the use of ^18^F-FDG PET/CT imaging SUVmax to assess the biological behavior of colon cancer is of great significance for guiding the choice of clinical treatment options.

This study also analyzed the relationship between the SUVmax of preoperative colon cancer primary lesions and the prognosis. The results showed that the 5-year event-free survival rate of the SUVmax > 18.26 group was significantly lower than that of the SUVmax ≤ 18.26 group. Therefore, the prognosis of colon cancer patients can be evaluated based on the SUVmax value of the primary tumor before surgery.

## 5. Conclusions

Exploring the correlation between preoperative ^18^F-FDG PET/CT imaging SUVmax of primary colon cancer and clinicopathological factors can guide the treatment and prognosis evaluation of colon cancer patients.

## Figures and Tables

**Figure 1:** Male, 69 years old. Sigmoid colon cancer lesions significantly uptake FDG (SUVmax, 37.6). The SUVmax of peri-intestinal metastases was about 8.4.

**Figure 2:** Female, 65 years old, colon cancer (SUVmax, 17.0). The SUVmax of enlarged lymph nodes beside the right colon (10 *∗* 11 mm) is about 4.6.

**Figure 3:** Male, 38 years old, having sigmoid colon cancer (SUVmax, 20.5) and multiple lung metastases (SUVmax, 15.3).

**Figure 4:** 5-year event-free survival rate.

**Table 1:** Clinicopathological information of 88 patients with colon cancer (*n*).

Group	*n*
Gender	
Male	52
Female	36
Age (year)	
<60	43
≥ 60	45
Tumor site	
Left colon	38
Right colon	50
Lesion length (cm)	I
<3	23
≥3	65
Pathological tissue type	
Mucinous adenocarcinoma	22
Adenocarcinoma	66
Tumor differentiation	
Well differentiated	21
Moderate differentiation	33
Poorly differentiated	34
AJCC stage	
0	2
I	4
II	16
III	22
IV	44

**Table 2:** Correlation analysis between the SUVmax value of ^18^F-FDG PET/CT imaging and clinicopathological factors before colon cancer surgery.

Group	n	SUVmax	T	*P* value
Gender			0.290	0.773
Male	52	16.38 ± 8.12^a^		
Female	36	15.32 ± 7.01		
Age (year)			0.283	0.775
<60	43	15.67 ± 6.89^a^		
≥60	45	15.79 ± 7.25		
Tumor site			0.501	0.623
Left colon	38	16.53 ± 8.01^a^		
Right colon	50	15.12 ± 7.32		
Lesion length (cm)			8.796	*P* ≤ 0.001^*∗∗*^
<3	23	9.12 ± 4.31^b^		
≥3	65	20.39 ± 9.63		
Clinical stage			7.863	*P* ≤ 0.001^*∗∗*^
0 + I + II	16	5.35 ± 2.67^b^		
III + IV	72	23.78 ± 9.02		
Pathological tissue type			10.356	*P* ≤ 0.001^*∗∗*^
Mucinous adenocarcinoma	22	8.75 ± 3.54^b^		
Adenocarcinoma	66	21.32 ± 9.76		
Tumor differentiation			9.265	*P* ≤ 0.001^*∗∗*^
Poorly differentiated	34	25.67 ± 12.31^b^		
Well and moderately differentiated	54	11.36 ± 5.06		

^*∗∗*^*P* ≤ 0.01.

**Table 3:** Comparison of results of clinical staging and pathological staging of 88 cases of colon cancer by 18 F-FDG PET/CT imaging.

PET/CT clinical stage	Postoperative pathological clinical stage					Sensitivity (%)	Specificity (%)	Accuracy (%)	PPV (%)	NPV (%)	Kappa	*P*
	0	I	II	III	IV							
I	2	4	0	0	0	100.0	97.6	97.7	66.7	100.0	0.788	<0.01
II	0	0	8	2	0	50.0	97.2	88.6	80.0	89.7	0.553	<0.01
III	0	0	8	20	0	90.1	87.9	88.6	71.4	97.1	0.722	<0.01
IV	0	0	0	0	44	100.0	100.0	100.0	100.0	100.0	100.0	<0.01

## Data Availability

The datasets used during the present study are available from the corresponding author upon reasonable request.
